The article "High Fat Diet Prevents Over-Crowding Induced Decrease of Sex Ratio in Mice" was published in 2011. Journal: PLoS One.

# High Fat Diet Prevents Over-Crowding Induced Decrease of Sex Ratio in Mice

**DOI:** 10.1371/journal.pone.0016296

**Published:** 2011-01-25

**Authors:** Madhukar Shivajirao Dama, Negi Mahendra Pal Singh, Singh Rajender

**Affiliations:** 1 Division of Endocrinology, Central Drug Research Institute (Council of Scientific and Industrial Research), Lucknow, India; 2 Biometry and Statistics Division, Central Drug Research Institute (Council of Scientific and Industrial Research), Lucknow, India; University of Dayton, United States of America

## Abstract

Adaptive theory predicts that mothers would be advantaged by adjusting the sex ratio of their offspring in relation to their offspring's future reproductive success. In the present study, we tested the effect of housing mice under crowded condition on the sex ratio and whether the fat content of the diet has any influence on the outcome of pregnancies. Three-week-old mice were placed on the control diet (NFD) for 3 weeks. Thereafter the mice were allotted randomly to two groups of 7 cages each with 4, 6, 8, 10, 12, 14, and 16 mice in every cage to create increasing crowding gradient and fed either NFD or high fat diet (HFD). After 4 weeks, dams were bred and outcomes of pregnancy were analyzed. The average dam body weight (DBW) at conception, litter size (LS) and SR were significantly higher in HFD fed dams. Further, male biased litters declined with increasing crowding in NFD group but not in HFD. The LS and SR in NFD declined significantly with increasing crowding, whereas only LS was reduced in HFD group. We conclude that female mice housed under overcrowding conditions shift offspring SR in favor of daughters in consistent with the TW hypothesis and high fat diet reduces this influence of overcrowding.

## Introduction

Trivers and Willard predicted that, the animals manipulate SR of their offspring when net fitness benefits conferred by investment in sons and daughters differ [1]. Regardless of their quality, daughters are more likely than sons to reproduce in many polygynous mating systems [2], [3]. Superior quality sons can leave many more offspring than daughters, but low-quality sons may fail to reproduce at all, making sons a more risky investment. Hence, in instances where the fitness gains of offspring quality are sex specific, a female in good condition (with ability to produce high-quality offspring) can be expected to produce more sons, whereas a female in poor condition (with no chances of producing high-quality offspring) will be expected to produce more daughters. Experimental evidence for biased offspring SRs gathered from many taxa supports this theory [reviewed in [4], [5]]. Numerous factors like maternal hormone levels [6], [7], [8], [9], [10], food abundance [11], [12], mate quality [13], habitat quality [14], dominance status [15], and maternal condition [16] influence the offspring SR. This hypothesis holds true for species with a small LS and depends on 3 assumptions [1]: 1) that the condition of the offspring at the end of the parental investment is correlated with the condition of the dam during parental investment; 2) that these differences in condition are carried over to adulthood; and 3) that the adult will be differentially advantaged in reproductive success through slight advantages in condition. Generally, any of the factors that have negative effects on mother favors female births and factors that have beneficial effects on mother favors male births. Even after accumulation of large amount of experimental support, the exact genetic and physiological basis for SR bias is still far from understood.

Despite consistent observations for many variables influencing maternal condition leading to SR variation considered individually, there are few studies reporting the influence of multiple factors [17]. Pratt and Lisk conducted two studies to show that dexamethasone and progesterone can prevent the SR deficit induced by social stress in golden hamsters [18], [19]. In the present study, we address one such problem by comparing the SR of two groups of mice (*Mus musculus*) that were maintained under increasing crowding conditions and fed either control diet (NFD) or high fat diet (HFD). Overcrowding is a most commonly employed method to produce a state of social stress in murine models [20], [21]. Supplementation of murine diet with slightly higher amount of dietary fat has been shown to increase the SR in mice [22], [23]. We hypothesized that overcrowding may decrease SR whereas HFD feeding should prevent the influence of overcrowding on SR.

## Results

The females on HFD had slightly lesser tendency to breed than females on NFD as 13 females failed to get pregnant in former as compared to 4 in latter. Data obtained from parallely running duplicate batches were used to replace for the failed pregnancies. There were no mortalities in either of the groups. Postnatal mortality of pups after second day of birth was higher in HFD (total 31 deaths) as compared to NFD (total 16 deaths). The DBW, LS and SR are summarized in Table 1.

**Table 1:** The summary (Mean ± SD) of dam body weight, litter size and sex ratio from NFD and HFD groups.

Variables	Crowdings	no of dams (n)	Diets	
			NFD	HFD
Dam body weight	1	4	20.25±2.06	22.65±1.28
	2	6	20.38±1.85	23.12±1.47
	3	8	21.15±1.88	22.51±2.34
	4	10	20.85±0.84	23.07±1.72
	5	12	21.26±1.33	22.83±1.45
	6	14	20.06±0.85	23.24±0.44
	7	16	21.21±1.28	22.85±1.65
*b*	*-*	*-*	*0.03, P = 0.53*	*0.02 P = 0.72*
Litter size	1	4	7.50±1.29	8.50±1.91
	2	6	8.17±0.75	8.67±1.03
	3	8	6.75±0.89	8.25±1.49
	4	10	7.20±1.23	8.40±0.70
	5	12	6.00±2.13	7.92±1.38
	6	14	5.14±0.66	6.29±1.14
	7	16	4.69±1.20	6.13±1.93
*b*	*-*	*-*	*−0.30, * ***P = 0.00***	*−0.26, * ***P = 0.00***
Sex ratio	1	4	0.52±0.14	0.50±0.07
	2	6	0.50±0.13	0.46±0.10
	3	8	0.49±0.15	0.53±0.14
	4	10	0.46±0.12	0.49±0.11
	5	12	0.42±0.20	0.52±0.17
	6	14	0.36±0.18	0.51±0.19
	7	16	0.31±0.18	0.49±0.27
*b*	*-*	*-*	*−0.02, * ***P = 0.00***	*0.001, P = 1.0*

The regression coefficient for rate of change in the variables with crowding is presented as *b*.

Comparing the effects of diet and crowding on DBW, LS, SR and proportion of male biased litters, ANOVA (Table 2) revealed a significant effect (*P*<0.01) of diet on DBW and LS, whereas crowding was found to have significant effect (*P*<0.01) on LS and proportion of male biased litters. However, the effect of diet, crowding and interaction of diet*crowding on SR was insignificant (*P*>0.05) (Table 2). Multiple comparison by Scheffe's post hoc test revealed that DBW at crowding 14 of NFD was significantly lower than crowding 14 of HFD (*P*<0.01), whereas there was no difference between groups for LS and SR.

**Table 2:** Analysis of variance summary for dam body weight, litter size, sex ratio and proportion of male biased litters from NFD and HFD groups.

Source of variation (SV)	Sum of squares (SS)	Degrees of freedom (DF)	Mean square (MS)	F-ratio	*P*-value
***Dam body weight***					
Diet	132.70	1	132.70	64.08	0.000
Crowding	4.71	6	0.78	0.38	0.891
Diet x Crowding	15.17	6	2.53	1.22	0.300
Error	260.95	126	2.07	-	-
Total	438.56	139	-	-	-
***Litter size***					
Diet	44.03	1	44.03	23.72	0.000
Crowding	165.63	6	27.60	14.87	0.000
Diet x Crowding	4.89	6	0.82	0.44	0.852
Error	233.84	126	1.86	-	-
Total	466.14	139	-	-	-
***Sex ratio***					
Diet	0.11	1	0.11	3.63	0.059
Crowding	0.21	6	0.04	1.13	0.346
Diet x Crowding	0.18	6	0.03	0.98	0.442
Error	3.95	126	0.03	-	-
Total	4.65	139	-	-	-
***Male biased litters***					
Diet	0.000	1	0.000	0.060	0.812
Crowding	0.006	6	0.001	16.54	0.002
Diet x Crowding	0.000	6	0.000	-	-
Error	0.000	0	-	-	-
Total	0.006	13	-	-	-

The mean DBW (22.93±1.48 vs. 20.80±1.37, t = 8.84; *P*<0.01), LS (7.39±1.73 vs. 6.06±1.69, t = 4.60; *P*<0.01) and SR (0.50±0.18 vs. 0.41±0.18, t = 2.96; *P*<0.01) for HFD group was significantly higher as compared to NFD. The SR was significantly lower in NFD compared to an expected value of 0.50 (t = 2.96, *P*<0.01), whereas it was unaffected in HFD (t = 0.00, P>0.05). The per cent male biased litters declined with increasing crowding in NFD group (from 50% in crowding 4 to 0% in crowding 16), whereas this parameter was almost similar in HFD group at all crowding levels. Overall, there were 16 male biased litters in NFD group and 29 in HFD group out of 70 litters in each (Figure 1).

**Figure 1:** Dam body weight at conception and outcomes of pregnancy in NFD and HFD groups. a) Dam body weight (b = 0.03 vs. 0.02, both *P*<0.05), b) Litter size (b = −0.30 vs. −0.26, both *P*<0.01), c) Percent male biased litters (b = −4.29, *P*<0.01vs. −0.36, *P*>0.05) and d) Sex ratio (*b* = −0.02, *P*<0.01 vs. 0.00, *P*>0.05). Squares represent NFD, crosses represent HFD, broken and solid lines are linear trends through NFD and HFD datasets, respectively.

Regressing sex ratio and male biased litters against crowding, regression analysis clearly showed that the SR and male biased litters in NFD declined significantly (*b* = −0.02 and −4.29; both *P*<0.01) while it was uniform at all the crowding in HFD (*b* = 0.00 and −0.36; both *P>*0.05). Similarly, with increasing crowding, the LS decreased significantly in both the diet groups (*b* = −0.30 and −0.26 for NFD and HFD respectively; both *P<*0.001). However, there was no change in DBW with increasing crowding in either group (*b* = 0.03 and 0.26 for NFD and HFD respectively; both *P*>0.05).

## Discussion

The decrease of SR with overcrowding is consistent with the adaptive sex allocation hypothesis of Trivers and Willard, in that female in poor condition; in this female under overcrowded condition produced more daughters than sons with fewer male biased litters. Further, prevention of the decrease of SR under overcrowding by feeding HFD can also be explained by the “better condition correlates with higher son births” explained in TWH. Several previous studies have shown that maternal stress due to any factor favor birth of daughters [18], [24], [25], [26], [27] and at least one study where housing mice under crowding condition produced a similar effect [28]. One report has established the SR increasing effects of diets enriched with fat in mice [22].

Housing laboratory animals under crowded conditions lead to various physiological effects producing a state of social stress due to increased competition for food, space and water [29]. Social stress favor female births as it ensures and increases reproductive success in female offspring who survive better than males both at embryonic and postnatal stages of life under limited resources availability [18], [24], [25], [28]. In case the overcrowding is affecting total food intake, it can explain the lower DBW in NFD. Alexenko et al., reported a similar effect on SR of pups born to mice while limiting the calorie intake by providing restricted amount of diet in mice [23]. Higher DBW in the HFD groups compared to NFD may be due to higher calorie availability with similar intake [22]. As the mice were given *ad libitum* access to feed throughout their lifetime, the crowding treatment represent a psychosocial stress treatment [30]. Similar to maternal body condition, various types of stressful stimuli acting around and/or after conception reduce the sex ratio in animals [18], [24], [25], [26], [27], [28], [31].

Our data suggest that LS may depend on both crowding and diet as it was comparable in both groups at lower crowding and decreased significantly with increasing crowding in both groups. The reduction in mean LS was evident earlier in NFD (i.e. at crowding 12) while evident late in HFD (i.e. at crowding 14) when compared to respective crowding 4. The mean male pup numbers in NFD also lowered significantly at crowding 14 and 16 as compared to crowding 4 while the same was not evident for female pups, number of male and female pups born to HFD dams did not change significantly with crowding. Social stress lead to smaller litters in mice and reduction of LS in both groups indicate that HFD cannot prevent effect of overcrowding on LS. Further, higher rate of reduction of male pup numbers (number of male biased litters was reduced drastically with each crowding) compared to female pup numbers at higher crowding in NFD suggest that male sex is more susceptible to overcrowding. ANOVA further confirmed this observation as crowding has a significant effect on the number of male biased litters.

The most striking observation from the present study was decline of SR with overcrowding and lack of this in HFD group. Unlike possible reduction in total calorie intake at higher densities in NFD, there appears to be no similar reduction in HFD groups as consumption of even lower quantity of HFD will supply more calories compared to NFD. Another possible physiological change that may be occurring is increased levels of circulating corticosteroid with overcrowding which leads to female favored births in some species [24]. Higher DBW during conception in HFD group can support overall higher SR but cannot explain the reduction specifically in NFD group with crowding as DBW was unaffected by crowding [23]. Further, the contribution of stud male on SR changes must also be negligible as they were all proven fertile males and exposed to the experimental diet for a very short period which is unlikely to change their X and Y sperm ratio [23]. Hence the only explanation for decreased SR in NFD group with crowding will be increased social stress. Even though we have not measured the systemic stress hormone levels, the correlation between cage density and stress is well established in mice. Since only difference between the two groups was the calorie density of diet, it can be concluded that HFD prevents overcrowding associated SR decrease in mice.

Like many other factors, social stress associated effects on sex ratios are believed to be non-adaptive as various studies have reported both male biased and female biased sex ratios in stressed animals [5], [32]. Considering this, the female biased sex ratios and reduced LS in crowded NFD dams and its prevention by HFD may be the outcome of physiological changes mediated through the influence of housing conditions and dietary fat without any adaptive significance. The dietary composition has myriads of effects on murine serum steroids, free fatty acid concentrations, vaginal pH, and induces molecular and physiological changes in the uterus [33], [34], [35].

In summary, we conclude that when female mice are housed under overcrowding conditions, they shift their offspring SR in favor of daughters and supplementation of diet rich in saturated fat containing higher calorie density reduces the influence of over-crowding. Though the mechanism by which the HFD reduces the influence of overcrowding on SR is not clear, we hypothesize that higher calorie intake may lead to such effect possibly by their ability to produce various physiological changes in the reproductive tract [23], [36] and providing a signal that environmental conditions are favorable. Recent findings have shown male embryos to be more sensitive to the drop in glucose levels than female embryos [37], [38]. Our study highlights the impact of simultaneous exposure to more than one potential variable affecting SR in mice and states that high fat diet could reduce female biased births under crowded conditions.

## Materials and Methods

### Ethics statement

All experiments were performed at the CDRI in accordance to the Institutional guidelines for the care and use of laboratory animals and were approved by the Institutional Animal Ethics Committee (IAEC approval number 25/09/ENDO/IAEC dated 19/01/2009), CDRI.

### Mice

Swiss albino mice were obtained from the inbred line maintained at the National Laboratory Animal Center (NLAC) of the Central Drug Research Institute (CDRI), Lucknow and housed at animal experiment unit under standard conditions.

### Diets

The control diet (NFD) and high fat diet (HFD) were procured from Tetragon Chemie Private Limited (TCPL), Bangalore, India. Lard was used as source of saturated fat to formulate the HFD. The TCPL provided the caloric and relative fat contents of two diets. The proportion of calories contributed by fat, carbohydrate and protein in NFD was 26%, 54%, and 20%, respectively while it was 58%, 22%, and 20%, respectively, in HFD. The energy density of NFD was 4.4 kcal/g while in HFD it was 4.8 kcal/g.

### Experimental setup

The aim of the present experiment was to compare the sex ratios of offspring born to dams that were housed in overcrowding condition and fed a Control diet (NFD) with those born to dams that were housed in overcrowding condition and fed the high fat diet (HFD). Age (21 days) and weight matched female mice (n = 140) were acclimatized to a 12 h day: 12 h night cycle for 3 wk, during which time they were fed the control diet. At the end of acclimation period, the mice were randomly divided into two diet groups (NFD and HFD, n = 70 each) with a further subdivision into 7 groups with each consisting of 4, 6, 8, 10, 12, 14 and 16 mice. All the mice in a subgroup were housed in a single cage so as to create increasing cage densities of 4 to 16 mice/cage. Polypropylene cages with floor area of 390 cm^2^ which can house 8 mice without leading to significant overcrowding (as per IAEC, CDRI) were used to house mice. Mice in both the groups were allowed *ad libitum* access to the diet. After completion of 4 weeks on experimental diets under gradient of crowding, dams were paired with stud males (aged ≈16 weeks), according to the protocol described by Rosenfeld et al. [22] On detection of copulatory plug, the females were weighed and transferred back to their respective cages. On completion of 17^th^ day after detection of vaginal plug, the pregnant females were separated and housed individually so that litters can be analyzed properly. Dams were observed four times daily form 18^th^ day of pregnancy to detect whelping and note the litter size (LS). Pups were sexed after 2 days of birth by measuring the ano-genital distance [39]. To confirm the accuracy of sexing method, genomic DNA was isolated from tail sample of 100 pups and analyzed by Polymerase chain reaction for the presence of SRY sequence (SRY is a male determining single copy gene located on Y chromosome) [40]. The complete experiment was conducted in duplicate to obtain data for cages with mice failing to breed, cannibalism, death or injury. Males were given *ad libitum* access to control diet, except during the mating period when they consumed the diet provided to females. Males were maintained on 12 h day and 12 h night cycle.

### Statistical analysis

The effect of two diets (NFD and HFD) and seven crowding levels (4, 6, 8, 10, 12, 14, 16) on dam body weight (DBW), LS and SR was analyzed separately by using general linear model (GLM) with factorial ANOVA and the significance of mean difference between groups was evaluated by Scheffe's post hoc test. Effect of diet and crowding on the proportion of male biased litters was analyzed by GLM with binomial distribution. DBW, LS and SR for the NFD and HFD groups were tested using a t-statistic. DBW and LS were compared between groups whereas SR was tested against an expected value of 0.5. The change in DBW, LS and SR within group with increasing crowding was analyzed using linear least square fitting (*b*). A two tailed (*α* = 2) probability (P) value <0.05 was considered to be statistically significant. All the statistical analysis was performed using STATISTICA (version 7.0).
